# Incidence, histopathologic analysis and distribution of tumours of the hand

**DOI:** 10.1186/1471-2474-15-182

**Published:** 2014-05-28

**Authors:** Maciej JK Simon, Pia Pogoda, Felix Hövelborn, Matthias Krause, Jozef Zustin, Michael Amling, Florian Barvencik

**Affiliations:** 1 Department of Osteology and Biomechanics, University Medical Center Hamburg-Eppendorf, Martinistr. 52, 20246 Hamburg, Germany; 2 Institute of Pathology, University Medical Center Hamburg-Eppendorf, Martinistr. 52, 20246 Hamburg, Germany

**Keywords:** Hand, Tumours, Histopathology, Incidence, Radiography

## Abstract

**Background:**

The aim of this large collective and meticulous study of primary bone tumours and tumourous lesions of the hand was to enhance the knowledge about findings of traumatological radiographs and improve differential diagnosis.

**Methods:**

This retrospective study reviewed data collected from 1976 until 2006 in our Bone Tumour Registry. The following data was documented: age, sex, radiological investigations, tumour location, histopathological features including type and dignity of the tumour, and diagnosis.

**Results:**

The retrospective analysis yielded 631 patients with a mean age of 35.9 ± 19.2 years. The majority of primary hand tumours were found in the phalanges (69.7%) followed by 24.7% in metacarpals and 5.6% in the carpals. Only 10.6% of all cases were malignant. The major lesion type was cartilage derived at 69.1%, followed by bone cysts 11.3% and osteogenic tumours 8.7%. The dominant tissue type found in phalanges and metacarpals was of cartilage origin. Osteogenic tumours were predominant in carpal bones. Enchondroma was the most commonly detected tumour in the hand (47.1%).

**Conclusions:**

All primary skeletal tumours can be found in the hand and are most often of cartilage origin followed by bone cysts and osteogenic tumours. This study furthermore raises awareness about uncommon or rare tumours and helps clinicians to establish proper differential diagnosis, as the majority of detected tumours of the hand are asymptomatic and accidental findings on radiographs.

## Background

Bone tumours are neoplasms originating in the skeletal system that are within or closely related to the bone tissue [1]. Primary bone tumours only account for a very small part of all human neoplasms and the bones of the hand are even more seldom affected [2,3]. The majority of tumours found in the hand are benign and of chondrogenic origin [3-5]. Almost all tumour types originating in bone can appear in the hand [6]. There have been numerous case reports of several tumour types of the hand [7-11], however, there is still a substantial lack of knowledge with regards to frequency and demographic knowledge about tumours of the hand.

The current article presents a large collection of hand tumours and demographic analyses. The aim of this meticulous study was to enhance the knowledge of findings on traumatological radiographs and improve differential diagnosis. Therefore, a comprehensive retrospective investigation was undertaken to characterise hand tumours and identify demographic and anatomic prevalence to aid the clinician.

## Methods

This retrospective study reviewed data collected from 1976 until 2006 in the Bone Tumour Registry Hamburg. The following data was documented: age, sex, radiological investigations, tumour location, histopathological features including type and dignity of the tumour, and diagnosis. The study was approved approval by the institutional ethics committee of the University Medical Center Hamburg-Eppendorf, Germany.

The tumours had been collected by our institution and from consultation cases sent to our Bone Tumour Registry. For all cases, undecalcifed specimens were embedded in methyl-methacrylate and/or embedded in paraffin wax after EDTA-decalcification. For the purposes of the present study, new fresh cut slides were prepared and stained with hematoxylin and eosin (paraffin blocks), or toluidine blue and Goldner trichrome staining methods (plastic embedded blocks). Microscopic analyses were done using a Zeiss microscope (Axiophot, Carl Zeiss, Jena, Germany) and representative microphotographs were taken using a digital camera (AxioCam MRc, Carl Zeiss, Jena, Germany) and AxioVision Rel.4.8. (Carl Zeiss, Jena, Germany).

Radiographs were collected for all cases included in this study.

All cases with osseous metastases, haematologic malignancies and inflammatory processes were excluded. The filtering process was executed and differentiation into five major tumour type categories was done as recommended by the World Health Organization (WHO) according to cell origin and one blend category was created and defined as “other” [12].

### Statistical analysis

For the statistical analysis, we used the global chi-squared test for analysis of sampling distribution with IBM® SPSS® Statistics 19. Significance was defined as p ≤ 0.05 and/or when p ≤ 0.01.

## Results

The retrospective analysis included 631 patients from 1976 until 2006 who met the inclusion criteria of a primary bone tumour confirmed by histopathologic analysis and not an osseous metastases, an inflammatory processes or of haematologic origin. The mean age was 35.9 ± 19.2 years. The distribution of tumour lesions in the right and left hand was 53.4 and 46.6 percent, respectively. The numbers of cases for each decade with additional separation by gender are illustrated in Figure 1 (Part A). The distribution by decade was significant according to the global chi-squared test. The gender break down revealed nearly equal occurrences: 50.7% for men and 49.3% for women (Figure 1B). Only 10.6% of all the registered tumours in our study were malignant (Figure 1C). Significant proportioning was found in the tumour tissue type classes with the cartilage-derived tumours being most dominant (69.1%, Figure 1D).

**Figure 1:** **Primary bone tumours and tumourous lesions of the hand from the Bone Tumour Registry Hamburg from 1976 until 2006.** Distribution of all cases per age decade with gender break down **(A)**. Total of 320 tumour lesions were detected in men and 311 in women **(B)**. Malignancies were found in 10.6% of all cases with an average age of 53.6 ± 24.3 years. Benign tumours were usually detected in younger patients (average age 33.8 ± 17.4 years) **(C)**. Tumour lesions were divided into six groups: cartilage, bone cysts, osteogenic, vascular, fibrogenic and other tumours **(D)**. Breakdown of tumour lesions into anatomical sites and malignant cases found in the specific site **(E)**.

Table 1 clearly illustrates that cartilage tumours were the most commonly found tumour in the hand (69.1%) followed by bone cysts with 71 cases (11.3%) in this study. Osteogenic tumours were only detected in 8.7% (n = 55). Vascular tumours appeared 14 times (2.2%), followed by fibrogenic tumours in 6 cases (0.9%). Forty-nine cases of different tumour entities were grouped together under “other” tumours (7.8%). Significance was calculated with the global chi-square test for enchondromas and giant cell tumours.The majority of hand tumours were found in the phalanges (69.7%); of these 10.2% were not benign. Metacarpal bones were affected in 24.7%. Malignancy in metacarpals was found in 12.2%. The carpal bones were affected by primary tumours in 5.5% of cases and of these 8.6% were malignant (Figure 1E). Another distribution perspective of the three skeletal parts of the hand is illustrated in Figure 2. Cartilage tumours in the phalanges and the metacarpal bones were the most often registered tumour type, 74.5% and 64.7% respectively. Osteogenic tumours (34.3%) were the highest in the carpal bones, but these were closely followed by bone cysts (28.5%) and cartilage tumours (20.0%). There were no fibrogenic tumours detected in the metacarpals or carpals.The following Figures 3, 4 and 5 illustrate the most often-occurring tumour types in the hand which surpassed the 5% margin of all bone tumours of the hand in the current dataset. Each of the following six tumour types is presented with a radiographic and a histological image. Additionally, the tumour distributions in the three anatomical sites of the hand as well as the occurrence of this particular tumour across life decades are demonstrated. In Figure 3A-D, enchondroma is presented which is the most frequently occurring tumour of the hand. The radiograph shows a medullary lesion with sharp margins in the proximal phalangeal bone (Figure 3A). Histologically, one identifies at low magnification a typical hypocellular area with a blue-gray taint in the cartilaginous matrix. There is hardly any manifestation of enchondromas in the carpal region (Figure 3C). The peak occurrence is identified for the fourth and fifth decade (Figure 3D). The second most often-occurring tumour type of the hand is the chondrosarcoma (Figure 3E-H). It appears only in the phalangeal and metacarpal region of the hand (Figure 3G). The tumour has a greater occurrence in later stages of life (Figure 3H). A typical ballooned cystic expansion is demonstrated in the metacarpal bone, which is very representative in appearance for an aneurysmal bone cyst (ABC) (Figure 4A). ABCs predominately manifest in the first 40 years of life (Figure 4D). The osteoid osteoma is more often present in the first 4 decades of life and in approximately 60% in the phalangeal bones (Figure 4G-H). A significant predominance of the osteochondroma is demonstrated for the phalanges (85.7%, Figure 5C). The current dataset only shows osteochondroma to be diagnosed by the end of the sixth decade, primarily in the first 20 years, thereafter no cases were reported (Figure 5D). Benign parosteal osteochondromatous proliferations (BPOP), also known as Nora’s lesion, were primarily found in the phalanges (84.9%, Figure 5G). Radiographic appearance demonstrates a cortical attachment and increased focal calcification in the lesion of the proximal phalanx (Figure 5E). The histological image partially resembles an appearance of osteochondromas (Figure 5F). It consists of cancellous bone with irregular cartilaginous or fibrocartilaginous tissue.

**Table 1:** A complete list of all tumour lesions found in the hand divided into six categories

**Cartilage tumours - 69.1%**				**Vascular tumours - 2.2%**			
	**Cases**	**Percentage**	**Avg. Age**		**Cases**	**Percentage**	**Avg. Age**
Enchondroma	297	47.10%	36.8 ± 14.7	Hemangioma	6	1.00%	24.5 ± 13.4
Chondrosarcoma	53	8.40%	60.7 ± 19.8	Hemangiopericytoma	2	0.30%	24.7 ± 28.3
Osteochondroma	35	5.50%	16.9 ± 18.2	Angiosarcoma	2	0.30%	20.5 ± 2.1
Enchondromatosis	28	4.40%	28.8 ± 19.3	Lymphangioma	2	0.30%	34.0 ± 26.8
Periostal chondroma	12	1.90%	22.8 ± 17.0	Glomustumour	1	0.20%	70.0 ± 0
Chondromyxoid fibroma	6	1.00%	37.0 ± 16.1	Skeletal angiomatosis	1	0.20%	36.0 ± 0
Chondroblastoma	5	0.80%	23.2 ± 13.9				
**Bone cysts - 11.3%**				**Fibrogenic tumours - 0.9%**			
	**Cases**	**Percentage**	**Avg. Age**		**Cases**	**Percentage**	**Avg. Age**
Aneurysmal bone cyst	52	8.20%	56.1 ± 16.5	Synovialoma	2	0.30%	17.7 ± 10.6
Simple bone cyst	13	2.10%	32.5 ± 20.1	Fibromyxoma	2	0.30%	23.5 ± 7.0
Epidermoid cyst	6	1.00%	55.5 ± 15.9	Desmoplastic fibroma	1	0.20%	68.0 ± 0
				Fibroxanthoma	1	0.20%	38.0 ± 0
**Osteogenic tumours - 8.7%**				**Other - 7.8%**			
	**Cases**	**Percentage**	**Avg. Age**		**Cases**	**Percentage**	**Avg. Age**
Osteoid osteoma	37	5.80%	35.9 ± 17.2	NORA	33	5.20%	46.2 ± 19.9
Perimyositis ossificans	7	1.10%	54.3 ± 20.7	Giant cell tumour	10	1.60%	35.5 ± 16.7
Osteosarcoma	6	1.00%	28.0 ± 19.0	Ewing sarcoma	3	0.50%	13.6 ± 6.4
Osteoblastoma	3	0.50%	34.3 ± 7.6	Malignant lymphoma	1	0.20%	73.0 ± 0
Osteom	2	0.30%	46.5 ± 13.4	Eosinophilic granuloma	1	0.20%	1.0 ± 0
				Neurilemmoma	1	0.20%	21.0 ± 0

**Figure 2:** **Anatomical site distribution of the six tumour categories.** Cartilage tumours dominate in the phalanges and metacarpals. Carpals are mostly affected by tumours of osteogenic origin.

**Figure 3:** **Enchondroma (A-D) and Chondrosarcoma (E-H) tumour characteristics are displayed.** A radiographic image **(A)** of a typical enchondroma located in the proximal phalangx and its’ histological image with toluidine blue stain **(B)**. Part C shows the distribution of enchondromas in the hand. A slightly higher prevalence emerges for the fourth decade. Microscopically **(D)**, the tumour consists of lobulated hyaline cartilage proliferation without cellular atypia. Chondrosarcomas were only found in the phalanges or metacarpals **(G)**. Radiographic **(E)** and histological images (hematoxylin and eosin stain [HE]) **(F)** demonstrated a typical cartilage tissue not respecting the structural boundaries. A higher incidence rate was found from the sixth decade onwards. Chondrosarcoma was microscopically characterised by slight cellular atypia and invasive growth **(H)**.

**Figure 4:** **Tumour lesion characteristics for aneurysmal bone cysts and osteoid osteomas.** Radiographic image of an aneurysmal bone cyst (ABC) detected in the proximal part of the forth digit **(A)**. Histological investigation **(B)** revealed blood-filled cystic spaces and numerous osteoclasts and hemosiderophage within the cyst walls. Locations of ABCs in the hand identify phalanges as the site most affected **(C)**. Prevalence was mostly in the first four decades. **(D)**. An osteoid osteoma of the thumb is displayed radiographically **(E)**. Number of cases and their distribution are displayed in part **G**. Osteoid osteomas were mostly found in the second to fourth decade **(H)**. The tumours were characterised by cellular bone forming neoplasm without atypia **(F)**.

**Figure 5:** **Osteochondroma and Nora's lesion tumour characteristics.** An osteochondroma is displayed in the X-ray **(A).** Microscopic analysis showed typical hyaline cartilage cup and growth plate-like bone proliferation **(B)**. Most cases were found in phalangeal bones (30 cases) **(C)** and early in life, first two decades **(D)**. Nora’s lesions can be identified in the radiographic image **(E)** and irregular periosteal chondro-osseous proliferation with no atypia **(F)**. Nora’s lesions were most often found in the phalanges **(G)**. Distribution of Nora’s lesions for gender and age is illustrated in part **H**.

## Discussion

There have been several reports demonstrating case-reports or collectives of specific tumour types, however, in our opinion there is a deficit in establishing a proper differential diagnosis of tumour lesions of the hand [10,13,14]. Therefore, this study included all types of primary tumours located in the hand. This systematic retrospective analysis of the collected data from the Bone Tumour Registry in Hamburg yielded a total of 631 cases divided into five major tissue types and one compilation of various tissue origins. Cartilage-derived tumours represented the main majority of all tumours of the hand. Furthermore, a predominance of tumours occurring in the phalanges was noted and the demographic distribution was significant aiding in establishing differential diagnoses.

A previous collection by Baumhoer and Jundt assembled chondrosarcomas, osteosarcomas and Ewing sarcomas and their main differential diagnoses [3]. Thus, their focus was on malignant tumours. They had registered 37 malignant bone tumours of the hands in the Basel Bone Tumour Reference Center since 1972 and reported clinical symptoms and presented valuable images.

However, there were more frequent tumour lesions than the ones listed by these authors. Therefore, we included in this current collection with over 600 cases all types of tumours found in the hand. Kitagawa and colleagues acknowledged the need to assess even soft-tissue tumours of the hand as there are bone changes associated with it [15]. They identified that many tumours are frequently associated with bone erosions. The erosions tend to increase in depth without increasing in width and often only require surgical curettage but bigger lesions require greater surgical approach.

In agreement with previous studies, benign tumours are significantly more common than malignant tumours in the hand [2,16-18]. Furthermore, elderly patients are more likely to have a malignant lesion whereas younger individuals present with a benign tumour. Enchondroma is the most common primary tumour lesion of the hand in the present study and as documented previously [19,20]. Enchondromas are benign but tend to have high cellularity, enlarged nuclei and double-nucleated cells making differentiation between benign tumours and malign lesions like chondrosarcomas difficult. However, proper diagnostic work up is essential to not miss any malignancies and determine accurate diagnosis followed by successful treatment. Chondrosarcomas were reported to metastasise and hence have the potential to be fatal [21]. Treatment of enchondromas is usually customised to the patient’s symptoms and risk for a pathologic fracture. Another tumour entity, which is special, is the bizarre parosteal osteochondromatous proliferation also known as Nora’s lesion, which is usually encountered on the surfaces of bones in hands and feet [13,22]. It has a relatively high recurrence rate between 29 to 55% [22,23]. It usually has a characteristic clinical and histologic appearance but still may be mistaken with other benign and malignant lesions like parosteal osteosarcoma. Though Nora’s lesions present with high recurrence rates and atypical histologic appearances, no metastases or deaths were reported, but high recurrence rates are indicative of a more extensive required resection in the treatment protocol [24,25].

The present study has several limitations. The study is retrospective and lacks clinical management, however; we believe that this was beyond the scope of our study. Additionally, the therapeutic regimens have changed considerably over the last decades. Furthermore, to have seen such an enormous collection of individuals and therefore to have personally gained differential diagnostic knowledge about tumour lesions of the hand is rather uncommon making this study tremendously valuable for the clinical practitioner. The cut-off mark for demonstrating the major tumour lesions was set at 5% covering over 80% of all lesions detected in the current study, and therefore should deliver sophisticated and at the same time not overwhelming advice for clinical practitioners.

## Conclusions

In conclusion, all primary skeletal tumours can be found in the hand and are most often of cartilage origin followed by bone cysts and osteogenic tumours. Phalanges of the hand most frequently have tumour lesions with enchondromas being the most often detected tumour overall. Additionally, two age peaks were identified for diagnosing tumour lesions of the hand: the second and forth decade. Over the observed time period of 30 years, malignant tumours were identified in about 11% of all cases and more often in older patients than benign lesions. These statistically evaluated results represent data of paramount importance for the clinician to help differentiate between various tumour entities in unclear, accidental or challenging radiographic findings with the use of the current data sets for tumour location, patient age and gender. Additionally, this research provides awareness of uncommon and rare tumours of the hand. Therefore, this information is extremely beneficial for the clinician in order to establish correct diagnosis early and consequently initiate proper treatment processes.

## Competing interests

The authors declare that they have no competing interests.

## Authors’ contributions

MJKS carried out the study’s concept design, data acquisition, data analysis, manuscript writing, and final approval. PP carried out the study’s concept design, data analysis, manuscript writing and revising, and final approval. FH participated in data acquisition and final approval. MK participated in data analysis and final approval. JZ participated in data acquisition, manuscript revising, and final approval. MA carried out the study’s concept design, data analysis, and final approval. FB carried out the study’s concept design, data analysis, manuscript writing and revising, and final approval.

## Pre-publication history

The pre-publication history for this paper can be accessed here:

http://www.biomedcentral.com/1471-2474/15/182/prepub
